# IL-17A promotes the neuroinflammation and cognitive function in sevoflurane anesthetized aged rats via activation of NF-κB signaling pathway

**DOI:** 10.1186/s12871-018-0607-4

**Published:** 2018-10-20

**Authors:** Zhan-yun Yang, Chang-xiu Yuan

**Affiliations:** Department of Anesthesia Surgery, Jining NO.1 People’s Hospital, No.6, Jiankang Road, Rencheng District, Jining, 272000 Shandong China

**Keywords:** Sevoflurane, IL-17A, NF-κB pathway, Neuroinflammation, Cognitive function

## Abstract

**Background:**

To investigate the role of IL-17A in the neuroinflammation and cognitive function of aged rats anaesthetized with sevoflurane through NF-κB pathway.

**Method:**

The aged and young adult rats were randomly divided into Control (inhale oxygen only), Sevoflurane (inhale oxygen and sevoflurane), Sevo (Sevoflurane) + anti-IL-17A (injected with IL-17A antibody, inhale oxygen and sevoflurane), and Sevo + NC groups (injected with IgG2a antibody, inhale oxygen and sevoflurane). Cognitive function was evaluated by Morris water maze and contextual fear conditioning tests. Tumor necrosis factor (TNF)-α, Interleukin (IL)-1β, IL-6 and monocyte chemoattractant protein (MCP)-1 expressions in the hippocampus of rats were detected by ELISA (enzyme-linked immunosorbent assay) assay, and Nuclear factor (NF)-κB pathway-related proteins by Western blot.

**Results:**

Sevoflurane anaesthetized aged rats showed longer escape latency and swimming distance, fewer platform crossing times, shortened stay time in the platform quadrant compared to Control rats; In addition, increased levels in hippocampal expression of malondialdehyde (MDA), IL-17A, NF-κB p65, inducible nitric oxide synthase (iNOS) and COX-2, as well as a reduced level of superoxide dismutase (SOD) were also observed in these animals. However, the sevoflurane anesthetized aged rats treated with anti-IL-17A presented a completely opposite tendency concerning the above factors (all *P* < 0.05). Nevertheless, there was no significant difference in the acquisition of learning or memory, neuroinflammation and oxidative stress of young adult rats in all groups (all *P* > 0.05).

**Conclusion:**

Anti-IL-17A may alleviate neuroinflammation and oxidative stress via inhibiting NF-κB pathway, thereby attenuating post-operative cognitive dysfunction (POCD) in aged rats anaesthetized with sevoflurane.

## Background

Postoperative cognitive dysfunction (POCD) refers to patients’ significant reduction in mental activity, personality, social activities and cognitive ability after anesthesia [1], which directly affects the quality of patients’ life and poses a great burden on patients’ family and the society [2]. Thus, reducing the incidence rate of POCD is of great importance for the clinical anesthesia and operation management. In recent years, anesthesia methods and the use of anesthetics have been suggested to be closely related to the occurrence of POCD [3]. Sevoflurane, as one of the most commonly used inhalation anesthetics in clinical practice, may induce mental retardation in children or trigger a higher incidence of POCD in elderly patients, when it inhaled in high concentrations or for many times [4, 5]. Besides, previous evidence has published that the major neurotoxicity of sevoflurane included the accumulation of β-amyloid protein (Aβ) [6], neuroinflammation [7], and reduction of synaptic plasticity [8], which have been accepted as the physiological basis of POCD in certain patients. At the same time, sevoflurane can stimulate the expression of inflammatory factors (like TNF-α and IL-1β) to induce neuroinflammation and neuronal damage, and thereby contributing to POCD [9, 10].

As a new cytokine, IL-17A is the first identified member belonging to the IL-17 family (IL-17A-F) [11], which could induce the secretion of pro-inflammatory cytokines, such as IL-1β, IL-6, and TNF-α, to exacerbate inflammatory responses [12], thus participating in numerous inflammatory-related diseases, including multiple sclerosis (MS) [13], cerebral ischemia [14], and rheumatoid arthritis (RA) [15]. Specifically, the increased expression of IL-17 and IL-22 receptors were observed by Kebir H et al. in the blood-brain barrier endothelial cells (BBB-ECs) from multiple sclerosis (MS) lesions, whereas IL-17 receptor inhibitor significantly alleviated the inflammation damage of central nervous system, which suggested that the brain damage of MS patients was related to the involvement of IL-17 [16]. Notably, there possibly existed a similar pathological mechanism between POCD and AD, indirectly implying an important role of IL-17A in POCD [17]. Additionally, NF-κB is considered as a crucial downstream transcription factor of the IL-17A signaling pathway [18], and NF-κB pathway has been suggested to involve in many essential biological processes, such as immune inflammatory response and cell apoptosis [19]. Moreover, 2% sevoflurane inhalation for 5 h was found to activate the NF-κB pathway in aged rats, thereby promoting the production of inflammatory factors, and affecting the learning and memory of rats [20], which further highlighted the involvement of NF-kB pathway in the pathogenesis of cognitive impairment in rats induced by sevoflurane.

Hence, the objective of this study is undertaken to explore the possible role of IL-17A in the neuroinflammation and cognitive function of aged rats anesthetized with sevoflurane via NF-κB pathway, thereby providing a novel strategy for the prevention and treatment of cognitive dysfunction.

## Methods

### Ethics statement

All experimental procedures for animals were approved by the Institutional Animal Care and Use Committee of the First People’s Hospital of Jining city and comply with the *Guide for the Care and Use of Laboratory Animals* published by the National Institutes of Health (NIH Publication No. 85–23, revised 1996) [21].

### Establishment and grouping of model rats with sevoflurane-induced cognitive dysfunction

A total of 96 healthy male Wistar aged rats (aged: 18–20 months; weighing: 500–700 g) and 96 young adult rats (aged: 2–3 months; weighing: 180–230 g) purchased from Shanghai Laboratory Animal Research Center of the Chinese Academy of Sciences, were randomly divided into four groups respectively: Control group, Sevoflurane group, Sevo (Sevoflurane) + anti-IL-17A group and Sevo + NC group (*n* = 24 per each group). One week before sevoflurane induction, rats in each group performed Morris water maze task training. Rats in the Control group continuously inhaled 30% O2-enriched air, while rats in Sevoflurane group inhaled 3.6% sevoflurane (No. H20110714, Maruishi, Japan) along with 30% O2 for 6 h. Notably, rats in the Sevo + anti-IL-17A group and Sevo + NC group were injected intravenously with 1 μg/kg of IL-17A antibody (R&D Systems, Minneapolis, MN, USA) and IgG2a antibody (Abcam,Cambridge, UK) separately, and one hour later, they continuously inhaled 3.6% sevoflurane with 30% O2 for 6 h. Twenty-four hours after anesthesia with sevoflurane inhalation, 8 rats were randomly selected from each group were killed by decapitation and the rat brain was quickly dissected. Then the hippocampus was quickly removed and homogenized in 100 mg/ml RIPA Lysis Buffer (Shenergy Biocolor Co., China) with 1% (*v*/v) PMSF (Shenergy Biocolor Co., China). The homogenate was centrifuged at 13 000 g for 20 min at 4 °C, and the supernatant was separated and stored at − 80 °C for further use. The other resting 16 rats in each group were not sacrificed and randomly used to conduct the Morris water maze test (*n* = 8) and Fear conditioning test (*n* = 8).

### Morris water maze test

The cognitive function of rats in each group were evaluated by using the Morris water maze test 24 h after anesthesia, which lasted for the first four days on place navigation test, and the fifth day on a spatial probe test. Rats were released into the water facing the wall from desired start point of the pool, and the time required to find the fixed platform (escape latency) was recorded. Rats should be kept on the platform for 30 s. If they failed to find the platform in 90 s, they should be led to the platform and stay there for 30 s. On the fifth day, the platform was taken out of the water, and rats were placed into the water from the former location. Then, the platform crossing times and the stay time in the platform quadrant were recorded.

### Fear conditioning test

Based on the procedures in a previous study [22], fear conditioning (FC) system was applied for the contextual fear conditioning memory test. One day before operation, rats were received the tone cued conditioning training. Next, rats were placed in experimental box for 2 min of adaption before giving them a continuous 70 dB sonic stimulation for 20 s (conditioned stimulus). Rats were given 0.7 mA foot shock for 2 s (unconditioned stimulus) 25 s after sonic stimulation. The procedures were repeated for six times at the interval of 60 s and the percentage of freezing time was recorded. On the 1st, 3rd and 7th day after anesthesia, the fear conditioning memory test was performed. In the contextual test, rats were placed in the box completely the same as the environment where they received electric shock, but they were not given sound and electric shock there. The percentage of time spent freezing (within 5 min) was recorded. In the tone cued test, the wallpaper in the conditional reaction box was replaced to change the environment. Then, rats were placed in there for 2 min of adaption and given continuous 70 dB sonic stimulation for 300 s, without electric shock. The percentage of time spent freezing should also be recorded.

### ELISA (enzyme-linked immunosorbent assay) assay

The hippocampal tissues (30 mg) were obtained from rats in each group, made into 10% hippocampal homogenate with normal saline, and centrifuged for 15 min at the rate of 5000 rpm. Then, the supernatant was collected and the ELISA kits (Wuhan Boster Biological Technology., LTD) were employed to detect the levels of TNF-α, IL-1β, IL-6 and MCP-1 in hippocampal tissues of rats. The contents of MDA and SOD in the hippocampus were measured by following the instructions on the ELISA kits.

### Western blot

The hippocampal tissues (20 mg) were mixed with 100–200 μl lysate, homogenized by a glass homogenizer, and centrifugated for 15 min at 12000 rpm. After collecting the supernatant, Sodium dodecyl sulphate-polyacrylamide gel electrophoresis (SDS-PAGE) was performed to separate proteins, which were transferred to the nitrocellulose membrane and blocked in 5% skim milk-PBS solution for 1 h at room temperature. Subsequently, primary antibodies were added for overnight incubation at 4 °C, including NF-κB p65 antibody (ab207297), iNOS antibody (ab15323), COX-2 antibody (ab15191), and IL-17A antibody (ab9056) (all diluted in 1:1000, Abcam). After the membrane rinsed with PBS buffer for three times, the secondary antibody crosslinked with HRP was added for 1 h of incubation at room temperature. At last, the membrane was washed with PBS buffer and enhanced chemiluminescence method was used for visualization. With β-actin as the internal reference protein, the gray value ratio of target band to reference band was regarded as the relative expression level of proteins.

### Statistical method

Statistical analysis was conducted by using the software SPSS 21.0. Measurement data were presented by mean ± standard deviation ($\overline{x}$± s). Differences between two groups were compared by using the Student’s t-test. One-Way ANOVA was used to analyze statistical differences among multiple groups and Tukey’s HSD test was used for post hoc testing. *P* < 0.05 indicated the statistical significance.

## Results

### Anti-IL-17A alleviated the cognitive impairment of sevoflurane-anaesthetized rats

As shown in Fig. 1, the ANOVA with Tukey’s HSD post hoc analysis demonstrated that exposure to sevoflurane in aged rats (Fig. 1a-d) enhanced escape latency (*F* = 116.4, *P* < 0.001) and swimming distance (*F* = 56.65, *P* < 0.001), decreased platform crossing times (*F* = 41.65, *P* < 0.001), and shortened stay time in the platform quadrant (*F* = 39.54, *P* < 0.0001). In addition, aged rats in the Sevo + NC group showed no significant difference in those indexes by comparison with in the Sevoflurane group (all *P* > 0.05), but anti-IL-17A reduced the escape latency and swimming distance, and increased platform crossing times and stay time in the platform quadrant in sevoflurane-anaesthetized rats (all *P* < 0.05), showing that anti-IL-17A could alleviate the cognitive impairment of aged rats after anesthesia with sevoflurane. Additionally, no significant difference was found in the escape latency (*F* = 0.775, *P* = 0.516), swimming distance (*F* = 2.148, *P* = 0.098), platform crossing times (*F* = 1.839, *P* = 0.163) and stay time in the platform quadrant (*F* = 0.531, *P* = 0.665) among groups of young adult rats (Fig. 1e-h).

**Fig. 1:** Comparison of the escape latency, swimming distance, platform crossing times and stay time in the platform quadrant of aged (**a**, **b**, **c**, **d**) and young adult (**e**, **f**, **g**, **h**) rats in each group. Note: Compared with the Control group, *, *P* < 0.05,**, *P* < 0.01, ***, *P* < 0.001; compared with the Sevoflurane group #, *P* < 0.05, ##, *P* < 0.01, ###, *P* < 0.001

### Comparison of fear conditioning memory test in rats

In both contextual (*F* = 139.3, *P* < 0.001) and tone cued fear conditioning sessions (*F* = 178.1, *P* < 0.001), significant differences among groups of aged rats were observed as displayed in Fig. 2a, b. The post hoc analysis showed that the aged rat in Sevoflurane group was significantly lower in the percentage of freezing time during contextual test and tone cued test on the 1st, 3rd and 7th day when compared to those in Control group (all *P* < 0.05). On the contrary, the aged rats in the Sevo + anti-IL-17A group had markedly higher percentage of freezing time in contextual test and tone cued test on the 1st, 3rd and 7th day after anesthesia than those in the Sevoflurane group (all *P <* 0.05), but there was no significant difference between the aged rats in Sevoflurane group and Sevo + NC group (all *P* > 0.05). Sevoflurane treatment had no effects on the percentage of freezing time during contextual test (*F* = 0.3007, *P* = 0.825) and tone cued test (*F* = 0.935, *P* = 0.428) in young adult rats as measured by ANOVA analysis (Fig. 1c, d).

**Fig. 2:** The percentage of freezing time at different time points after anesthesia in each group. Note: **a**, **b** The percentage of freezing time at different time points of contextual test and tone cued test of aged (**a**, **b**) and young adult (**c**, **d**) rats in each group. Compared with the Control group, *, *P* < 0.05,**, *P* < 0.01, ***, *P* < 0.001; compared with the Sevoflurane group #, *P* < 0.05, ##, *P* < 0.01, ###, *P* < 0.001

### Levels of inflammatory factors of rats in each group

The ANOVA with Tukey’s HSD post hoc analysis shown that the levels of inflammatory factors, including TNF-α (*F* = 282.4, *P* < 0.001), IL-1β (*F* = 199.2, *P* < 0.001), IL-6 (*F* = 169.9, *P* < 0.001) and MCP-1 (*F* = 172.4, *P* < 0.001) were remarkably increased in the hippocampus of aged rats in the Sevoflurane group as compared with the Control group (Fig. 3a). At the same time, compared with those in the Sevoflurane group, the aged rats in the Sevo + NC group showed no significant difference in the above inflammatory factors (all *P* > 0.05), whereas those in the Sevo + anti-IL-17A group had apparently reduced levels of TNF-α, IL-1β, IL-6 and MCP-1 (all *P* < 0.05). Nevertheless, there was no significant difference in the levels of TNF-α (*F* = 1.768, *P* = 0.176), IL-1β (*F* = 0.653, *P* = 0.588), IL-6 (*F* = 0.591, *P* = 0.626) and MCP-1 (*F* = 2.133, *P* = 0.118) among the four groups of young adult rats (Fig. 3b).

**Fig. 3:** The expression levels of TNF-α, IL-1β, IL-6 and MCP-1 in the hippocampus of aged (**a**) and young adult (**b**) rats in each group detected by ELISA. Note: Compared with the Control group, *, *P* < 0.05,**, *P* < 0.01, ***, *P* < 0.001; compared with the Sevoflurane group #, *P* < 0.05, ##, *P* < 0.01, ###, *P* < 0.001

### Comparison of contents of MDA and SOD in the hippocampus of rats in each group

We found significant group differences of aged rats in the MDA (*F* = 231.3, *P* < 0.001) and SOD content (*F* = 63.15, *P* < 0.001) as illustrated in Fig. 4a. For all of these main effects, post hoc analyses revealed that exposure to sevoflurane in aged rats resulted in increased MDA content and decreased SOD content as compared to Control group (all *P* < 0.05). However, the decreased MDA content and increased SOD content were observed in the hippocampus of aged rats in the Sevo + anti-IL-17A group as compared to Sevoflurane group (all *P* < 0.05), and no statistical difference was found between the Sevoflurane group and the Sevo + NC group in the hippocampal MDA and SOD contents (all *P* > 0.05). There was no significant difference in the MDA (*F* = 1.192, *P* = 0.331) and SOD (*F* = 0.142, *P* = 0.934) contents of young adult rats in all groups (Fig. 4b).

**Fig. 4:** Comparison of the contents of MDA and SOD in the hippocampus of aged (**a**) and young adult (**b**) rats in each group. Note: Compared with the Control group, *, *P* < 0.05,**, *P* < 0.01, ***, *P* < 0.001; compared with the Sevoflurane group #, *P* < 0.05, ##, *P* < 0.01, ###, *P* < 0.001

### Expression of IL-17A and NF-κB pathway-related proteins of rats in each group

The ANOVA with Tukey’s HSD post hoc analysis indicated that the protein expressions of IL-17A (*F* = 186.5, *P* < 0.001), NF-κB p65 (*F* = 167.7, *P* < 0.001), iNOS (*F* = 237.3, *P* < 0.001) and COX-2 (*F* = 168.8, *P* < 0.001) increased statistically in the hippocampus of aged rats in the Sevoflurane group. Besides, no statistical difference in these proteins was observed between the aged rats in Sevoflurane group and Sevo + NC group (all *P* > 0.05), but the aged rats in the Sevo + anti-IL-17A group had decreased expressions of IL-17A, NF-κB p65, iNOS and COX-2 when compared to Sevoflurane group (all *P* < 0.05, Fig. 5a). There was no significant difference in the protein expressions of NF-κB p65 (*F* = 1.900, *P* = 0.1526), iNOS (*F *= 2.384, *P* = 0.091) and COX-2 (*F* = 2.630, *P* = 0.070) of young adult rats in all groups. However, the ANOVA analysis shown the protein expressions of IL-17A was significantly reduced in the Sevo + anti-IL-17A group (*F *= 38.19, *P* < 0.001, Fig. 5b).

**Fig. 5:** Comparison of expressions of IL-17A and NF-κB pathway-related proteins of aged (**a**) and young adult (**b**) rats in each group. Note: Compared with the Control group, *, *P* < 0.05,**, *P* < 0.01, ***, *P* < 0.001; compared with the Sevoflurane group #, *P* < 0.05, ##, *P* < 0.01, ###, *P* < 0.001

## Discussion

As reported, the Morris water maze test is widely applied in behavioral performance to evaluate spatial learning and memory ability in mazes on animals, which has been extensively used in the investigation of the related neurocognitive disorders [23]. To be specific, the place navigation test shown as an elevation in escape latency indicate the decline in the cognitive ability of spatial memory [24], while the increased platform crossing times and target-quadrant stay time reflect better-consolidated spatial information ability in general proficiency and strategies use [25]. In addition, the fear conditioning memory model has gradually become an important leading behavioral model for studying the neurobiological mechanism of learning and memory owing to its relatively accurate and stable text results [26, 27]. As such, we evaluated the cognitive function of rats by the Morris water maze test and fear conditioning memory test, and the aged rats induced by using 3.6% sevoflurane for 6 h presented the prolonged escape latency and swimming distance, decreased platform crossing times and the percentage of stay time on the target-quadrant, as well as the reduced percentage of time spent freezing in the fear memory test, indicating that inhalation of 3.6% sevoflurane for 6 h can induce cognitive impairment in aged rats. Hu et al. in his study also found the similar concentration of sevoflurane could disrupt the integrity of blood-brain barrier of aged rats to induce cognitive impairment [28]. Notably, there was evidence showing that desflurane anesthesia was dependent on dose, which resulted in significant impairment of acquisition learning and memory of aged rats with the higher dose of 3.6% desflurane exposure [29]. But 4 h of 2.4% sevoflurane exposure did not impair acquisition learning and retention memory in both young adult and aged rats in the study by Callaway JK et al. [30]. However, the cognitive function of young adult rats was not influenced by sevoflurane exposure in our observations, which was consistent with the findings of Callaway JK and the colleague. Furthermore, sevoflurane did not significantly increase hepatic injury in the young male rats, but caused more hepatic injury in old rats, as illustrated by Arslan M et al. [31]. Thus, we may suggest that the effect of sevoflurane anesthesia on acquisition learning or memory in rats are age and dose dependent. Besides, the normal function of hippocampus has been reported to be necessary for the formation and retrieval of memory in aversive conditioning such as contextual fear conditioning [32]. While the deficits observed in contextual freezing may be due to hippocampal deficits, and the amygdala impairment can be responsible for disrupting freezing responses to tone cues [33]. In our study, the aged and young adult rats were also to have a decreased freezing to both contextual and tone conditioning over time (1d, 3d, and 7d). Most importantly, the altered hippocampus functioning in rats was confirmed in the passive avoidance test where the consolidation of contextual fear memories appeared to be time-limited [34]. Similar to consolidation, reconsolidation also requires new protein synthesis and has a limited time window of approximately several hours after memory reactivation [35]. Altogether, these findings point out the possibility that, the decreased freezing over time may depend on the extinction of memory in rats on the 3rd and 7th day in the fear conditioning.

More importantly, anti-IL-17A treatment significantly improved results in the Morris water maze test and the fear memory test in the anesthetized aged rats. There was also evidence revealed that blocking IL-17 can reduce the cognitive impairment caused by surgical trauma-induced inflammation via regulation of TGF-β/Smad pathway and the expression of Aβ1–42 [36], suggesting that anti-IL-17A treatment can significantly alleviate the cognitive function of aged rats anesthetized with sevoflurane.

Besides, we also detected the indicators related to oxidative stress and inflammatory factors in rats, probably since the induction of POCD by sevoflurane has close relations with the increased oxidative stress and inflammatory factors in the central nervous system, such as TNF-α and IL-1β [37]. As shown by the results in our study, the levels of inflammatory factors (TNF-α, IL-1β, IL-6 and MCP-1) of aged rats were remarkably elevated in sevoflurane-anesthetized rats, with the increased MDA and reduced SOD content. Nevertheless, exposure to sevoflurane had no significant effect on any of the levels of inflammatory factors, as well as MDA and SOD content in young adult rats. As previously demonstrated, the immune inflammatory response in the central nervous system is mainly mediated by activated glial cells and the release of inflammatory mediators [38]. Specifically, activated glial cells could secrete a large amount of pro-inflammatory factors, like IL-1β, TNF-α and IL-6, and in turn, IL-1β could bind to receptors on the membrane to further activate glial cells and release more cytokines, which constituted a positive feedback of inflammation cascade reaction to accelerate Aβ deposition and neuronal apoptosis, thereby inducing neurotoxicity and cognitive dysfunction [10, 39, 40]. In agreement, Lu et al. also showed Aβ protein accumulation and increased inflammatory mediators in the central nervous system in neonatal mice after the sevoflurane anesthesia [41]. On the other hand, oxidative stress, mainly induced by free radicals and disrupted oxidative defense system, is considered as an important pathophysiological basis of various aging-related degenerative diseases, since superoxide radicals produced during this process could cause damage to the brain tissues and promote the aging and death of brain cells [42, 43]. Of note, MDA levels could reflect the degree and severity of cellular injury [44], while SOD, a scavenger of superoxide, presented the antioxidant capacity [45]. In this study, anti-IL-17A treatment resulted in the reduced levels of inflammatory factors and inhibited oxidative stress, suggesting that anti-IL-17A may improve the cognitive function of anesthetized aged rats by reducing neuroinflammation and oxidative stress.

Furthermore, the expression of downstream NF-κB signaling pathway of IL-17A was determined in our research. As a consequence, the expression levels of IL-17A, NF-κB p65, iNOS and COX-2 increased significantly in the hippocampus of rats in the Sevoflurane-induced aged rats, but not in young adult rats. The up-regulation of NF-κB and IL-6 was also measured by Zhang et al. in glial cells after anesthesia with isoflurane and sevoflurane, which was very likely to be related to the learning and cognitive function after anesthesia [7], but declined statistically after the treatment with anti-IL-17A, suggesting that anti-IL-17A can inhibit NF-κB pathway in the hippocampal tissues of anesthetized aged rats. Another precious study has stated that IL-17 can promote the binding of Act1 (an activator of NF-κB) and IL-17R via the interaction of SEFIR-SEFIR domains, to induce the activation of downstream signal NF-κB [46]. When nerve tissues damaged, IκB kinase (IKK) would be activated to induce phosphorylation of IκB, and then NF-κB dimers would enter the cell to recognize promoters of IL-6 and TNF-α, promote transcription of inflammatory factors, ultimately activating the inflammatory reaction [47, 48]. Apart from that, ROS produced during oxidative stress can inhibit the release of IκB and activate NF-κB, thereby inducing the transcription of downstream cytokines iNOS and COX-2 [49, 50]. Meanwhile, the activated iNOS could produce the synthesis of a large number of NO, which would be toxic to neural cells and cause cell death [51, 52]. Consistent with our study, IL-17A can activate NF-κB and P13K/Akt signal transduction pathways in Hwang et al.’s experiment, to induce the production of IL-6 and IL-8 by synovial fibroblasts in RA patients [53]. Moreover, anti-IL-17 significantly reduced the expression of NF-κB in asthmatic mice, contributing to inhibition of the expression of inflammatory factors, the remodeling of extracellular matrix, and oxidative stress [54]. Interestingly, our study found that anti-IL-17A in the young rats decreased IL-17A but did not affect the expression levels of NF-κB, iNOS and COX-2, which may be attributed to the differences in NF-κB pathway levels between aged rats and young adult rats when exposed to sevoflurane. In particular, anti-IL-17A might decrease NF-κB pathway levels in sevoflurane-treated aged rats to a level sufficient to restore normal function, but did not change the expressions of sevoflurane-treated young adult rats which had originally normal levels of NF-κB pathway.

## Conclusions

In sum, we come to a conclusion that anti-IL-17A treatment may improve neuroinflammation and oxidative stress by inactivation of NF-κB pathway, eventually alleviating cognitive impairment of aged rats with sevoflurane anesthesia.

## References

[1] Hovens IB, Schoemaker RG, van der Zee EA, Absalom AR, Heineman E, van Leeuwen BL (2014). Postoperative cognitive dysfunction: involvement of neuroinflammation and neuronal functioning. Brain Behav Immun.

[2] Postoperative cognitive dysfunction (2005). Rev Bras Anestesiol.

[3] Jungwirth B, Zieglgansberger W, Kochs E, Rammes G (2009). Anesthesia and postoperative cognitive dysfunction (POCD). Mini reviews in medicinal chemistry.

[4] Xia Y, Xu H, Jia C, Hu X, Kang Y, Yang X, Xue Q, Tao G, Yu B (2017). Tanshinone IIA attenuates sevoflurane neurotoxicity in neonatal mice. Anesth Analg.

[5] Purdon PL, Pavone KJ, Akeju O, Smith AC, Sampson AL, Lee J, Zhou DW, Solt K, Brown EN (2015). The ageing brain: age-dependent changes in the electroencephalogram during propofol and sevoflurane general anaesthesia. Br J Anaesth.

[6] Zhang B, Tian M, Zheng H, Zhen Y, Yue Y, Li T, Li S, Marcantonio ER, Xie Z (2013). Effects of anesthetic isoflurane and desflurane on human cerebrospinal fluid Abeta and tau level. Anesthesiology.

[7] Zhang L, Zhang J, Yang L, Dong Y, Zhang Y, Xie Z (2013). Isoflurane and sevoflurane increase interleukin-6 levels through the nuclear factor-kappa B pathway in neuroglioma cells. Br J Anaesth.

[8] Haseneder R, Kratzer S, von Meyer L, Eder M, Kochs E, Rammes G (2009). Isoflurane and sevoflurane dose-dependently impair hippocampal long-term potentiation. Eur J Pharmacol.

[9] Rosczyk HA, Sparkman NL, Johnson RW (2008). Neuroinflammation and cognitive function in aged mice following minor surgery. Exp Gerontol.

[10] Vacas S, Degos V, Feng X, Maze M (2013). The neuroinflammatory response of postoperative cognitive decline. Br Med Bull.

[11] Iwakura Y, Ishigame H, Saijo S, Nakae S (2011). Functional specialization of interleukin-17 family members. Immunity.

[12] Ma X, Reynolds SL, Baker BJ, Li X, Benveniste EN, Qin H (2010). IL-17 enhancement of the IL-6 signaling cascade in astrocytes. J Immunol.

[13] Balasa R, Bajko Z, Hutanu A (2013). Serum levels of IL-17A in patients with relapsing-remitting multiple sclerosis treated with interferon-beta. Mult Scler.

[14] Zhang J, Mao X, Zhou T, Cheng X, Lin Y (2014). IL-17A contributes to brain ischemia reperfusion injury through calpain-TRPC6 pathway in mice. Neuroscience.

[15] Hueber AJ, Asquith DL, Miller AM, Reilly J, Kerr S, Leipe J, Melendez AJ, McInnes IB (2010). Mast cells express IL-17A in rheumatoid arthritis synovium. J Immunol.

[16] Kebir H, Kreymborg K, Ifergan I, Dodelet-Devillers A, Cayrol R, Bernard M, Giuliani F, Arbour N, Becher B, Prat A (2007). Human TH17 lymphocytes promote blood-brain barrier disruption and central nervous system inflammation. Nat Med.

[17] Li ZG, Zhang W, Sima AA (2007). Alzheimer-like changes in rat models of spontaneous diabetes. Diabetes.

[18] Ivanov S, Linden A (2009). Interleukin-17 as a drug target in human disease. Trends Pharmacol Sci.

[19] Zhang G, Liu R, Zhong Y, Plotnikov AN, Zhang W, Zeng L, Rusinova E, Gerona-Nevarro G, Moshkina N, Joshua J (2012). Down-regulation of NF-kappaB transcriptional activity in HIV-associated kidney disease by BRD4 inhibition. J Biol Chem.

[20] Tian Y, Guo S, Wu X, Ma L, Zhao X (2015). Minocycline alleviates sevoflurane-induced cognitive impairment in aged rats. Cell Mol Neurobiol.

[21] Bayne K. Revised guide for the care and use of laboratory animals available. American Physiological Society The Physiologist. 1996;39(4):199 208-111.8854724

[22] Vizcaychipi MP, Xu L, Barreto GE, Ma D, Maze M, Giffard RG (2011). Heat shock protein 72 overexpression prevents early postoperative memory decline after orthopedic surgery under general anesthesia in mice. Anesthesiology.

[23] Del Rosario Adeline, McDermott Mindy M., Panee Jun (2012). Effects of a high-fat diet and bamboo extract supplement on anxiety- and depression-like neurobehaviours in mice. British Journal of Nutrition.

[24] Baldi E, Efoudebe M, Lorenzini CA, Bucherelli C (2005). Spatial navigation in the Morris water maze: working and long lasting reference memories. Neurosci Lett.

[25] Snihur AW, Hampson E, Cain DP (2008). Estradiol and corticosterone independently impair spatial navigation in the Morris water maze in adult female rats. Behav Brain Res.

[26] Hobin JA, Goosens KA, Maren S (2003). Context-dependent neuronal activity in the lateral amygdala represents fear memories after extinction. J Neurosci.

[27] Cole CJ, Mercaldo V, Restivo L, Yiu AP, Sekeres MJ, Han JH, Vetere G, Pekar T, Ross PJ, Neve RL (2012). MEF2 negatively regulates learning-induced structural plasticity and memory formation. Nat Neurosci.

[28] Hu N, Wang C, Zheng Y, Ao J, Zhang C, Xie K, Li Y, Wang H, Yu Y, Wang G (2016). The role of the Wnt/beta-catenin-Annexin A1 pathway in the process of sevoflurane-induced cognitive dysfunction. J Neurochem.

[29] Callaway JK, Jones NC, Royse AG, Royse CF (2015). Memory impairment in rats after desflurane anesthesia is age and dose dependent. J Alzheimers Dis.

[30] Callaway JK, Jones NC, Royse AG, Royse CF (2012). Sevoflurane anesthesia does not impair acquisition learning or memory in the Morris water maze in young adult and aged rats. Anesthesiology.

[31] Arslan M, Ozkose Z, Akyol G, Barit G (2010). The age- and gender-dependent effects of desflurane and sevoflurane on rat liver. Exp Toxicol Pathol.

[32] Nasuti C, Fattoretti P, Carloni M, Fedeli D, Ubaldi M, Ciccocioppo R, Gabbianelli R (2014). Neonatal exposure to permethrin pesticide causes lifelong fear and spatial learning deficits and alters hippocampal morphology of synapses. J Neurodev Disord.

[33] Laurent V, Westbrook RF (2010). Role of the basolateral amygdala in the reinstatement and extinction of fear responses to a previously extinguished conditioned stimulus. Learn Mem.

[34] Gafford GM, Parsons RG, Helmstetter FJ (2011). Consolidation and reconsolidation of contextual fear memory requires mammalian target of rapamycin-dependent translation in the dorsal hippocampus. Neuroscience.

[35] Yang C, Liu JF, Chai BS, Fang Q, Chai N, Zhao LY, Xue YX, Luo YX, Jian M, Han Y (2013). Stress within a restricted time window selectively affects the persistence of long-term memory. PLoS One.

[36] Tian A, Ma H, Zhang R, Tan W, Wang X, Wu B, Wang J, Wan C (2015). Interleukin17A promotes postoperative cognitive dysfunction by triggering beta-amyloid accumulation via the transforming growth factor-beta (TGFbeta)/Smad signaling pathway. PLoS One.

[37] Zheng JW, Meng B, Li XY, Lu B, Wu GR, Chen JP (2017). NF-kappaB/P65 signaling pathway: a potential therapeutic target in postoperative cognitive dysfunction after sevoflurane anesthesia. European review for medical and pharmacological sciences.

[38] Santa-Cecilia FV, Socias B, Ouidja MO, Sepulveda-Diaz JE, Acuna L, Silva RL, Michel PP, Del-Bel E, Cunha TM, Raisman-Vozari R (2016). Doxycycline suppresses microglial activation by inhibiting the p38 MAPK and NF-kB signaling pathways. Neurotox Res.

[39] Pan Y, Chen XY, Zhang QY, Kong LD (2014). Microglial NLRP3 inflammasome activation mediates IL-1beta-related inflammation in prefrontal cortex of depressive rats. Brain Behav Immun.

[40] Zhang YY, Fan YC, Wang M, Wang D, Li XH (2013). Atorvastatin attenuates the production of IL-1beta, IL-6, and TNF-alpha in the hippocampus of an amyloid beta1-42-induced rat model of Alzheimer's disease. Clin Interv Aging.

[41] Lu Y, Wu X, Dong Y, Xu Z, Zhang Y, Xie Z (2010). Anesthetic sevoflurane causes neurotoxicity differently in neonatal naive and Alzheimer disease transgenic mice. Anesthesiology.

[42] Paradies G, Petrosillo G, Paradies V, Ruggiero FM (2011). Mitochondrial dysfunction in brain aging: role of oxidative stress and cardiolipin. Neurochem Int.

[43] Uttara B, Singh AV, Zamboni P, Mahajan RT (2009). Oxidative stress and neurodegenerative diseases: a review of upstream and downstream antioxidant therapeutic options. Curr Neuropharmacol.

[44] Baierle M, Nascimento SN, Moro AM, Brucker N, Freitas F, Gauer B, Durgante J, Bordignon S, Zibetti M, Trentini CM *et al*: Relationship between inflammation and oxidative stress and cognitive decline in the institutionalized elderly. Oxidative Med Cell Longev 2015, 2015:804198.10.1155/2015/804198PMC438340325874023

[45] Zhang K, Zhang Q, Jiang H, Du J, Zhou C, Yu S, Hashimoto K, Zhao M (2018). Impact of aerobic exercise on cognitive impairment and oxidative stress markers in methamphetamine-dependent patients. Psychiatry Res.

[46] Liu C, Swaidani S, Qian W, Kang Z, Sun P, Han Y, Wang C, Gulen MF, Yin W, Zhang C (2011). A CC' loop decoy peptide blocks the interaction between Act1 and IL-17RA to attenuate IL-17- and IL-25-induced inflammation. Sci Signal.

[47] Guo F, Xing Y, Zhou Z, Dou Y, Tang J, Gao C, Huan J (2012). Guanine-nucleotide exchange factor H1 mediates lipopolysaccharide-induced interleukin 6 and tumor necrosis factor alpha expression in endothelial cells via activation of nuclear factor kappaB. Shock.

[48] Kumar A, Negi G, Sharma SS (2012). Suppression of NF-kappaB and NF-kappaB regulated oxidative stress and neuroinflammation by BAY 11-7082 (IkappaB phosphorylation inhibitor) in experimental diabetic neuropathy. Biochimie.

[49] Kim H, Youn K, Ahn MR, Kim OY, Jeong WS, Ho CT, Jun M (2015). Neuroprotective effect of loganin against Abeta25-35-induced injury via the NF-kappaB-dependent signaling pathway in PC12 cells. Food Funct.

[50] Qi S, Xin Y, Guo Y, Diao Y, Kou X, Luo L, Yin Z (2012). Ampelopsin reduces endotoxic inflammation via repressing ROS-mediated activation of PI3K/Akt/NF-kappaB signaling pathways. Int Immunopharmacol.

[51] Yu HH, Wu FL, Lin SE, Shen LJ (2008). Recombinant arginine deiminase reduces inducible nitric oxide synthase iNOS-mediated neurotoxicity in a coculture of neurons and microglia. J Neurosci Res.

[52] Mander P, Brown GC (2005). Activation of microglial NADPH oxidase is synergistic with glial iNOS expression in inducing neuronal death: a dual-key mechanism of inflammatory neurodegeneration. J Neuroinflammation.

[53] Hwang SY, Kim JY, Kim KW, Park MK, Moon Y, Kim WU, Kim HY (2004). IL-17 induces production of IL-6 and IL-8 in rheumatoid arthritis synovial fibroblasts via NF-kappaB- and PI3-kinase/Akt-dependent pathways. Arthritis research & therapy.

[54] Camargo LDN, Righetti RF, Aristoteles L, Dos Santos TM, de Souza FCR, Fukuzaki S, Cruz MM, Alonso-Vale MIC, Saraiva-Romanholo BM, Prado CM, et al. Effects of anti-IL-17 on inflammation, remodeling, and oxidative stress in an experimental model of asthma exacerbated by LPS. Front Immunol. 2017;8:1835.10.3389/fimmu.2017.01835PMC576051229379497

